The article "Structural Design and Preliminary Tests of a Novel Patient Transfer Apparatus for Medical Scenarios" was published in 2021. Journal: J Healthc Eng.

# Structural Design and Preliminary Tests of a Novel Patient Transfer Apparatus for Medical Scenarios

**DOI:** 10.1155/2021/2770846

**Published:** 2021-08-03

**Authors:** Yu Tian, Hongbo Wang, Yongshun Zhang, Bowen Su, Jiazheng Du, Xincheng Wang, Yongfei Feng, Bo Cheng, Jianye Niu

**Affiliations:** ^1^Parallel Robot and Mechatronic System Laboratory of Hebei Province, Yanshan University, Qinhuangdao 066004, China; ^2^Academy for Engineering & Technology, Fudan University, Shanghai 200433, China; ^3^Faculty of Mechanical Engineering & Mechanics, Ningbo University, Ningbo 315211, China; ^4^Operating Room, Qinhuangdao Hospital of Traditional Chinese Medicine, Qinhuangdao 066004, China; ^5^Key Laboratory of Advanced Forging & Stamping Technology and Science of Ministry of Education, Yanshan University, Qinhuangdao 066000, China

## Abstract

Patient transfer has always been a difficult problem, usually requiring multiple caregivers to work together, which is time consuming and can easily cause secondary injuries to the patient. In addition, with the crisis of COVID-19, the issue of patient transfer is even more critical, as caregivers are at a high risk of infection, causing significant damage to healthcare resources. In this paper, a patient transfer assist system named E-pat-plus (Easy Patient Transfer plus) has been proposed; it can assist caregivers in transferring patients, reduce direct contact between them, and avoid secondary injuries. In the mechanical structure of this apparatus, a novel five-gear assembly module and a synchronous belt pulley set are proposed; they are the key points to the basic functional realization of the device and can reduce the cost of the prototype. Furthermore, a fuzzy (proportion-integration-differentiation) PID-based cross-coupling control strategy is applied to the apparatus to ensure the stability and safety of the operation. Finally, some preliminary experiments, including current experiments and error experiments, are carried out to verify the reliability of the device and lay the foundation for clinical tests.

## 1. Introduction

At present, research on the causes and diagnostic methods of COVID-19 has achieved significant results, and vaccines have been developed and are being rolled out around the world [1–3]. However, the global epidemic situation is still not promising. During the treatment of COVID-19, the patient transfer is an unavoidable process (e.g., between wards, operating rooms, and ICU) in which doctors and caregivers must prevent themselves from being infected. Although medical protective clothing can play an effective role in protection, too much contact with the patients is bound to increase the probability of being infected, and this adds tremendous psychological pressure to doctors and caregivers. In fact, the infection could cause great damage to the healthcare system and impose a serious burden on society [4]. Therefore, it is a meaningful research topic to reduce the infection rate during the transfer process by using advanced robotic systems.

Research on patient transfer-assisted systems has been conducted for some time [5–7]. Initially, caregivers used bed sheets and soft boards as media to transfer patients between beds. This was based on human labor and the continuous work would cause damage to the caregivers [8]. Therefore, some automated transfer equipment has been gradually developed. At present, according to the form of equipment, it can be divided into four types: belt type, flat plate type, chair/bed type, and humanoid type.

Among them, the belt type uses flexible straps to carry patients by lifting, and the straps can be fixed on the ceiling moving device [9] or the floor moving device [10, 11]. This type of equipment is flexible; multiple patients can share one single device, and it will not be limited by the bed layout during usage. The core components of the flat plate type are thin plates and belts [12, 13], which work on the principle of relative motion between objects. When the device moves close to the patient, the belts rotate in reverse on the surface of the plate, so there exists no significant relative movement between the patient and the bed in the horizontal direction, and there is only a small change in height, thus achieving a safe and smooth transfer process of the patient. The chair/bed type is a combination of a bed and a wheelchair; it usually consists of a U-shaped bed and a foldable wheelchair [14–16]. This type of equipment integrates the functions of the bed and wheelchair, and they have the advantages of higher transfer efficiency and less physical/mental burden on the patients. The humanoid type can be divided into two forms of embracing robots and bearing robots: the former generally contains two robotic arms, and the latter has one more chest support plate than the former. This type usually has more degrees of freedom [17, 18] and can also improve the perception of the environment by installing sensors [19]. Currently, simplified versions of the aforementioned devices have been applied to the market [20–24].

Although all the aforementioned devices can transfer patients and effectively reduce the direct contact between caregivers and patients, there are differences in the scope of application and other aspects. Specifically, the belt type can pick up the patient regardless of the size and weight of the user, but the patient is required to have the ability to sit on his own. The flat plate type allows the patient to complete the transfer process in a lying posture, which is very suitable for users who have almost lost the ability to move, but there are two difficulties. The first is to solve the contradiction between the design of the ultrathin mechanism and the motor arrangement, and the second is the coordination work of the motors. The solution to these two problems is beneficial to improve the comfort for the users. The chair/bed type is safer and more versatile, but it costs much more because one device can be used by only one patient. In addition, the separate design of the bed and wheelchair makes it difficult to arrange the bed sheet. The humanoid type has more degrees of freedom and requires a certain level of moving mobility for the user, and it usually costs more than the chair/bed type.

For patients suffering from COVID-19, their respiratory system is severely impaired, and complications lead to a reduction in their ability to move. Therefore, the following principles should be satisfied when using robots to transport patients with COVID-19: (1) the contact frequency between caregivers and patients can be significantly reduced; (2) patients who have almost lost the ability to move can also be transferred; (3) the change in patients' posture during the transport process should be as small as possible to avoid secondary injuries. Among all the aforementioned devices, only the flat plate type and the chair/bed type have these characteristics. The number of patients with COVID-19 is large, and each chair/bed robot can be used by only one person, which is inefficient and costly; therefore, the flat plate type is probably the best choice. Based on our team's existing research [25], a new flat-type device has been proposed that can satisfy the design principles above, and some fresh ideas have been proposed in this paper.

This paper proposed a novel patient transfer-assisted system named E-pat-plus (see Figure 1), which is a flat plate-type device that has a double-layer structure that completes the transfer process through the synchronous movement of pulleys and belts, reducing the contact frequency between caregivers and patients. The power of this device is provided by a symmetrically arranged power module, which adapts to the physiological curvature of the human body and reduces the pressure on the cervical spine, playing the role of a “pillow.” This device enables the user to maintain a lying position when transferring, and the angle of the sagittal plane for the users changes less, so patients with little motion ability can be easily transferred by this device. This device adopts a fuzzy PID-based cross-coupled synchronous control strategy to ensure comfort, and it can be remotely controlled, which can also reduce the risk of infection for caregivers.

The rest of this paper is organized as follows. The innovative design of the mechanical structure is introduced in Section 2. The control strategy of the device is proposed in Section 3, and a comparison of the synchronous control strategy is proposed.  Section 4 shows the preliminary tests of E-pat-plus, which proves the reliability of the prototype.  Section 5 gives the conclusion and future work.

## 2. Innovative Design of E-Pat-Plus

E-pat-plus is a flat plate-type device and works on the principle of relative motion between objects; that is, for the upper and lower belts moving at speeds V and −V, respectively, the relative velocities of the objects on either side of them (here, the bed and the patient, respectively) are 0 (see Figure 2). This allows the patient's posture to remain constant during the transfer, ensuring patient safety and reducing the muscle strength required during the process.

E-pat-plus is modular in design and mainly includes the upper module, lower module, and power module (see Figure 3). The power module contains all the controllers, motors, and other driving components. This device is symmetrical from the internal composition. There are six flat belts on the surface of the upper module for lifting the patient, which is in direct contact with the patient throughout the working process; therefore, in addition to meeting the demand of the transfer function, the safety and comfort of the patient is also an important factor that should be taken into account. The lower module drives the device and the patient to move together, so it needs to have a strong bearing capacity and walking ability. The upper and lower modules complete the transfer process through cooperative motion and ensure that the patient's posture does not change significantly, avoiding secondary damage.

The upper module consists of two identical parts, one of which includes a motor, a five-gear assembly module, four synchronous belt pulley sets, flat belts, and so on (see Figure 4). To illustrate the working process of the upper module clearly, the pulley sets are named set 1, set 2, set 3, and set 4. The flat belts of the upper module are fixed with an open loop; i.e., the two ends of the belt are fixed to set 1 and 3 (or set 2 and 4), respectively, to realize the movement of the belt on the surface of the aluminum plate and complete the patient transfer when one set tightens the belt and the other releases. The open loop method has both advantages and disadvantages; it can avoid belt runout problems and requires less tensioning force. As a trade-off measure, the inability to perform continuous circular motion leads to complexity in mechanical design. In addition, the thickness of the belts at both ends is different during almost all the working processes, which makes it difficult to control the belt. To compensate for these shortcomings while reducing costs (i.e., using one motor), three innovative tips are proposed to solve the aforementioned problems. First, a synchronous belt pulley set has been designed as a flat structure that reduces the belt thickness of winding on the set in the initial position (at this time, the thickness is maximum); the second is to calculate the minimum length of the flat belt on the basis of satisfying the transfer process to further ensure that the thickness is the lowest; third, limit blocks have been arranged on the five-gear assembly module, using the distance (circumference) between the initial positions of the limit blocks to compensate for the difference in linear speed between the gears and the rollers. For the first point, the flat synchronous belt pulley set consists of the main beam, secondary beam, supporting screws, adjusting screws, synchronous belt, and rollers, wherein the main beam and secondary beam can slide relative to each other to facilitate the installation and tensioning. The supporting screws can fix the position of the two beams and the adjusting screws can ensure the parallelism of the two synchronous rollers. The advantages of the module are demonstrated by a comparison with cylindrical rollers, i.e., the total belt thickness is smaller on the flat structure when winding the same length of the belt. Regarding the second point, the installation length of the flat belt can be approximately equivalent to twice the width of the device, and the length of the belt motion while transferring the patient onto the device is also approximately equal to the width. In some cases, the equipment needs to drive a way from underneath the patient after the transfer process, and another width of the device is needed. The ultimate length requirement should be three times the width of the device. For the third point, the distribution of limit blocks is also shown in Figure 3, and the working principle is illustrated through a moving process. Assuming the drive gear rotates clockwise, the rotation direction of other gears and rollers is shown in Figure 3. At this time, all flat belts are wound on set 1 and set 3 is the active drive part. The belt thickness of the sets can be described as follows:

(1) $$\begin{array}{c} \left\{\begin{array}{c} A=2\times \left(a+\pi \cdot r_{1}\right),\\ B=\left[\frac{2S}{A}\right]+1, \end{array}\right. \end{array}$$

where *A* represents the perimeter of the synchronous belt pulley set, *a* is the center distance of the synchronous rollers, *r*_1_ is the radius of the rollers, *B* is the maximum number of turns of flat tape winding, and *S* is the width of the device. For the results of *B*, increment processing is adopted to ensure reasonableness. The gears on both sides are driven by one motor, so the angular speed is the same, and the linear speed of the rollers on both sides (the speed of the belt motion) is also the same. However, there are flat belts winding on the right synchronous belt pulley set, so on the right side, the roller rotates lower than the gear. At this time, the gear and roller on the left side move together, their limit blocks are pressed against each other, and the motion of the gear and roller on the right side is separate. Furthermore, in a complete transfer process, the limit block on the gear cannot “catch up” with the block on the roller, which guarantees continuous and safe work; thus, the dimensional constraints for the mechanism design can be obtained:

(2) $$\begin{array}{c} \frac{S}{2\pi \cdot r_{1}}-\frac{S}{2\pi \cdot \left(r_{1}+h\times \left(\left[S/A\right]+1\right)\right)}\leq 1, \end{array}$$

where *h* is the thickness of the flat belt; that is, when the movement distance is *S*, the number of turns for the gear is no more than 1 turn of the roller, so that the gear always moves at a position not more than one circumference in front of the roller in one movement cycle. When the moving distance is between *S* and 2*S*, this motion process is symmetrical with the previous motion process, the thickness of the left set is greater than that of the right set, and the angle speed of the right roller is faster than that of the gear, i.e., the roller slowly catches up with the gear again. In summary, the limit blocks on the gears and the roller will not interfere during all working conditions, and the transfer process is safe enough as long as the constraints are met.

The lower module is the chassis of E-pat-plus (see Figure 5), mainly composed of motors, travel modules, connecting rods, etc. Each travel module consists of brackets, active/passive synchronous pulleys, and synchronous belts. There are tensioning rollers on each side of the active synchronous pulleys, which not only has the function of tensioning but also increases the wrap angle to prevent the phenomenon of jumping teeth. Such tensioning rollers are arranged at both sides of the travel module to further ensure reliability. The passive pulleys at both ends have a higher axial position, the purpose of which is to guarantee the ability to cross obstacles, such as pressing forward over a warped bedsheet instead of being entangled with it. The lower module is directly connected to the frame by hexagonal bolts. Due to the limited space on both sides, the motor and external meshing gear sets are arranged on the side.

## 3. Control Strategy of E-Pat-Plus

### 3.1. Establishment of the Upper-Module Dynamic Model

During the operation of this device, the stability of the system is of great significance to the safety and comfort of the patient and must be considered. As mentioned before, E-pat-plus is divided into three mechanical modules, and a load of each module is different; therefore, the different motion speeds of the body parts during the transfer process are the main reason for the patient's discomfort. To solve this problem, the requirement for the device is to maintain the stability of the single motor and the synchronization of multiple motor movements for the upper module. This chapter models the dynamics of the upper module, and a fuzzy proportion-integration-differentiation (PID) control algorithm is proposed to eliminate the nonlinear uncertain factors in the system, which improves the accuracy and anti-interference ability of the motor. For the two motors in the upper module, three possible synchronization control strategies for this device have been explored, and simulations are performed and compared.

The power transmission process of the upper module is displayed (see Figure 6). The motor is connected to the driving gear, and the power is transmitted to the inner/outer gears through the five-gear assembly module. The inner gear drives the synchronous belt wheel, the synchronous belt, and the flat belt, in turn, thereby pulling the patient to move. The outer gear transmits the power to the head and foot drive rollers to drive the head/foot movement.

According to the movement process, ignoring the influence of internal friction and the deformation and vibration of the synchronous belt during transmission, the dynamic equations of related parts are established in turn:

(3) $$\begin{array}{c} \left\{\begin{array}{c} T_{m}=J_{s}\frac{d^{2}\theta_{m}}{dt^{2}}+B_{s}\frac{d\theta_{m}}{dt}+J_{1}\frac{d^{2}\theta_{m}}{dt^{2}}+T_{1},\\ T_{1}=2J_{2}\frac{d^{2}\theta_{m2}}{dt^{2}}+2J_{3}\frac{d^{2}\theta_{m3}}{dt^{2}}+T_{2}+T_{3},\\ T_{2}=2\left(4J_{p1}\frac{d^{2}\theta_{p1}}{dt^{2}}+4J_{p2}\frac{d^{2}\theta_{p2}}{dt^{2}}+J_{x1}\frac{d^{2}\theta_{p1}}{dt^{2}}+J_{x2}\frac{d^{2}\theta_{p1}}{dt^{2}}\right)+F_{d1}\cdot r_{p1},\\ T_{3}=2\left(J_{p3}\frac{d^{2}\theta_{p3}}{dt^{2}}+J_{p4}\frac{d^{2}\theta_{p4}}{dt^{2}}+J_{p5}\frac{d^{2}\theta_{p5}}{dt^{2}}+J_{p6}\frac{d^{2}\theta_{p6}}{dt^{2}}\right)+F_{d2}\cdot r_{p3}, \end{array}\right. \end{array}$$

where *F*_*d*1_=*μm*_1_*g*=*m*_1_(d^2^*x*_*s*_/d*t*^2^) and *F*_*d*2_=*μm*_2_*g*=*m*_2_(d^2^*x*_*s*_/d*t*^2^) represent the friction generated by the load at both ends (head/foot), respectively; *x*_*S*_=*θ*_*p*1_ · *r*_*p*1_=*z*_1_/*z*_2_ · *r*_*p*1_ · *θ*_*m*_ represents the relationship between the position of the load and the rotation angle of the motor. Combining the above equations and bringing in the ratio relationship between the gears, the motor driving torque can be expressed as follows, and the symbols that are not described are shown in the table (see Table 1).

(4) $$\begin{array}{c} T_{m}=\frac{z_{2}}{z_{1}}\cdot \frac{1}{r_{p1}}\left(\begin{array}{c} J_{s}+J_{1}+2\cdot \frac{z_{1}}{z_{2}}\cdot J_{2}+2\cdot \frac{z_{1}}{z_{3}}\cdot J_{3}+8\cdot \frac{z_{1}}{z_{2}}\cdot J_{p1}\\ +8\cdot \frac{z_{1}}{z_{2}}\cdot \frac{r_{p1}}{r_{p2}}\cdot J_{p2}+2\cdot \frac{z_{1}}{z_{2}}\cdot J_{x1}+2\cdot \frac{z_{1}}{z_{2}}\cdot J_{x2}\\ +2\cdot \frac{z_{1}}{z_{3}}\cdot J_{p3}+2\cdot \frac{z_{1}}{z_{3}}\cdot \frac{r_{p3}}{r_{p4}}J_{p4}+2\cdot \frac{z_{1}}{z_{3}}\cdot \frac{r_{p3}}{r_{p5}}\cdot J_{p5}\\ +2\cdot \frac{z_{1}}{z_{3}}\cdot \frac{r_{p3}}{r_{p6}}\cdot J_{p6}+m_{1}\cdot \frac{z_{1}}{z_{2}}\cdot r_{p1}^{2}+m_{2}\cdot \frac{z_{1}}{z_{2}}\cdot r_{p1}\cdot r_{p3} \end{array}\right)\frac{d^{2}x_{s}}{dt^{2}}+\frac{z_{2}}{z_{1}}\cdot \frac{1}{r_{p1}}\cdot B_{s}\frac{dx_{s}}{dt}. \end{array}$$

### 3.2. Design and Simulation of Fuzzy PID Controller

Fuzzy PID is a combination of fuzzy control and the PID algorithm. Fuzzy control mainly consists of four steps, namely, fuzzification, rule base establishment, logic judgment, and defuzzification. The PID control strategy is a classic closed-loop control strategy that is widely adopted in industry and the laboratory. It is characterized by the ability to make timely adjustments to external changes, strong anti-interference ability, and fast response time. In this controller model, the input is the error *e* and the error rate of change *de*, which refer to the displacement error of the synchronous belt, and the output is the proportional coefficient *k*_*p*_, differential coefficient *k*_*d,*_ and integral coefficient *k*_*i*_. The initial values of the parameters are determined as *k*_*p*_ = 2.1, *k*_*i*_ = 1.8, and *K*_*d*_ = 0.42 by the engineering trial method. The value of the error fuzzy domain is [−4, 4], and the rate fuzzy domain is [−4, 4]. The basic domain of Δ*k*_*p*_ is [−0.6, 0.6], the basic domain of Δ*k*_*i*_ is [−0.11, 0.1], and the basic domain of Δ*k*_*d*_ is [−0.2, 0.2]. The language variables are set to 7 levels, namely, negative big, negative medium (NB), negative small (NS), zero (ZO), positive big (PB), positive medium (PM), and positive small (PS), and the triangular affiliation function is chosen as the affiliation function. The area center of gravity method is taken as the clear method.

A comparison model between traditional PID and fuzzy PID is built in a simulation environment, and the performance is analyzed. Due to the nonlinear and uncertain interference factors in the real environment, disturbances are added to the system. The response to a unit step signal is displayed (see Figure 7). It can be concluded that fuzzy PID can adjust parameters in real time to ensure that the system is in a relatively stable state so that the system can maintain good anti-interference under the condition of nonlinear and uncertain interference caused by more transmission components. The overshoot is smaller, and the error is smaller.

### 3.3. Analysis of the Synchronization Control Strategy

As mentioned before, the synchronous motion of the motors plays an important role in the comfort and safety of the patient. The upper module is driven by two motors; therefore, synchronization control algorithms need to be designed to maintain the synchronization of motor motion. At present, there are some mature methods to solve this problem. According to the functional requirements of the device, three possible effective strategies are initially considered: parallel synchronization control strategy, master-slave synchronization control strategy, and cross-coupling synchronization control strategy.

All the strategies are carried out based on the feedback of the encoder. A proMOTION brand motor is adopted in E-pat-plus. Its model is 36SYK62, and the rated voltage is 24 VDC, the rated current is 3.2 A, and the encoder resolution is 800 pulses. For the parallel synchronization control strategy, the motors receive the desired speed value at the same time, and the controller adjusts the speed in real time according to the feedback of the encoder to ensure the synchronization of the motor and the stability of the system. For the master-slave control strategy, the two motors are marked as the master motor and slave motor, and only the master motor receives the desired speed. The output speed of the master motor is used as the input speed of the slave motor; therefore, any speed change of the former is transmitted to the latter, thus ensuring synchronization of the motion. For cross-coupling control, the motors also receive the desired speed at the same time. In addition, a compensator is added to the feedback process, and the core of this compensator is to extract the difference between the output speed of the two motors and multiply it by certain factors. Then, the compensated speed is fed back to the motors to ensure synchronization. The basic mathematical expressions for the velocity and displacement errors are the same in the three methods and can be expressed as follows:

(5) $$\begin{array}{c} \left\{\begin{array}{c} \Delta \omega_{i}\left(t\right)=\omega_{s}\left(t\right)-\omega_{i}\left(t\right)\;\left(i=1,2\right),\\ \Delta \omega_{12}\left(t\right)=\omega_{1}\left(t\right)-\omega_{2}\left(t\right)=\Delta \omega_{2}\left(t\right)-\Delta \omega_{1}\left(t\right),\\ s=\int_{0}^{t}\Delta \omega_{12}\left(t\right)\text{d}t=\int_{0}^{t}\left[\Delta \omega_{2}\left(t\right)-\Delta \omega_{1}\left(t\right)\right]\text{d}t, \end{array}\right. \end{array}$$

where *ω*_*s*_(*t*) is the desired speed set from the host controller, *ω*_*i*_(*t*) represents the output speed of the motor, and *s* means the displacement error of the two motors, which is the integral of the velocity. Furthermore, the principle of the compensator in cross-coupling control is as follows:

(6) $$\begin{array}{c} \left\{\begin{array}{c} \omega_{f1}\left(t\right)=\omega \left(t\right)+k_{1}\left[\omega_{1}\left(t\right)-\omega_{2}\left(t\right)\right],\\ \omega_{f2}\left(t\right)=\omega \left(t\right)+k_{2}\left[\omega_{1}\left(t\right)-\omega_{2}\left(t\right)\right], \end{array}\right. \end{array}$$

where *ω*_*f*1_(*t*) and *ω*_*f*2_(*t*) are the compensated speeds of the motors, and *k*_1_ and *k*_2_ are the scale factors that generally take equal values in the symmetrical two-motor system. To select the most suitable control strategy for E-pat-plus, the aforementioned alternative methods are modeled in MATLAB/Simulink to compare their speed error and displacement error (see Figure 8). The input speed is 50 mm/s, which approximates the actual working speed, and the disturbance term is added to the system at 2 s due to the nonlinear interference in the transfer process.

The results are displayed (see Figure 9). In 0–2 s, the speed error of parallel synchronization control strategy and cross-coupling is zero when there is no disturbance in the system, and the error under the master-slave synchronization control strategy exhibits a sudden change at first and then rapidly reduces to zero. This is because the input of the slave motor originates from the master. In 2–6 s, the disturbance term is added and the speeds under the three methods can all maintain a small error, but the cross-coupling control strategy gives the smallest error. Regarding the displacement error of the system, within 0–2 s, there exists a sudden change in the error under the master-slave control strategy and the error under the parallel synchronous control strategy and the cross-coupling synchronous control strategy is zero. In 2–6 s, the displacements under the three methods can all maintain a small error, and the cross-coupling control strategy gives the smallest error. According to the analysis above, the cross-coupling control strategy has the best behavior, and the master-slave control strategy is the worst.

In the master-slave control strategy, the input of the slave motor is heavily dependent on the master, which is the reason for the large speed and displacement errors; therefore, its application effect is the worst in the work scene of E-pat-plus. The parallel synchronous control strategy can realize the closed-loop feedback of a single motor control loop, but the connection between the two motors is not close. For the cross-coupling control strategy, feedforward control is added, and the compensation speed of a single motor is related to the output speed of all motors, strengthening the connection between them so it has better performance. Therefore, the cross-coupling synchronization control strategy is finally selected.

## 4. Preliminary Experiments of E-Pat-Plus

### 4.1. Transfer Process of the Device

To demonstrate the performance of the equipment clearly, the transfer process and preliminary experiments of E-pat-plus are presented in this chapter. The process of transferring can be divided into four steps: approaching the patient, raising the patient, human-machine integrated movement, and completing the transit process (see Figure 10). In the first step, the flat belts on the upper module are stationary, and the synchronous belts on the lower module move separately. The device leaves the stretcher and lands on the bed. In the second step, the upper and lower modules move together to lift the patient onto the device, and the patient only has variations in the vertical position and a small amount of sagittal inclination, which makes him comfortable and safe. In the third step, the device works in the same state as the first step; the difference is that the movement of the synchronous belts on the lower module is reversed, i.e., the patient and the device return together from the bed to the stretcher. In the last step, the patient and the device arrive at the stretcher, and the transfer process is completed. After that, the patient can be transferred to other medical scenes (operating rooms, wards, examination rooms, etc.) by the stretcher. It can be seen from the working process that E-pat-plus can transfer patients automatically, and there is less contact between the caregiver and the patient, which greatly reduces the possibility of infection and physical burden for the caregiver. The task of caregivers has changed from contact load bearing to noncontact observation, that is, observation of the patient's state (expression, body motion, etc.) during the transfer process to ensure that safety is sufficient.

### 4.2. Preliminary Experimental Trial of E-Pat-Plus

Experiments on current and errors are conducted to test the load capacity and synchronization of the prototype in this part. During the experimental session, a laptop computer replaced the remote control as the host controller of the system to observe the value of the encoders. The rated load of E-pat-plus is 130 kg, and its weight is approximately 40 kg. To simulate the uneven weight distribution of the transfer process, blocks of 80 kg and 50 kg are arranged on the two upper modules, and the ratio of the mass blocks on the 3 belts of each module is 1 : 2 : 2; therefore, the weights of the masses on the 6 belts are 16 kg, 32 kg, 32 kg, 10 kg, 20 kg, and 20 kg. The device is turned over to perform tests on the lower module. Considering the mass distribution ratio of the upper module, the mass blocks equivalent to the self-weight of the device are equally distributed to the four synchronous belts, so the four synchronous belts have loads of 50 kg, 50 kg, 35 kg, and 35 kg.

In the current experiment, the currents of the individual motors in the upper and lower modules are tested separately under the aforementioned load conditions (see Figure 11). It can be observed that the maximum operating current of the four motors does not exceed the rated current, indicating that all the motors can still work in a safe state when the device is fully loaded; the average current of the upper module is 1.0 A, and the average current of the lower module is 1.4 A, which is in line with the actual situation in which the load of the lower module is greater than that of the upper module.

In the experiment of the errors, the effectiveness of the synchronization control algorithm was tested, and the errors of the upper and lower modules were examined with/without the synchronization control algorithm. It can be seen from the results (see Figure 12) that the speed error without the algorithm is approximately ±5 mm/s and is approximately ±2 mm/s with the algorithm during the movement of the upper module. The speed error without the algorithm is approximately −3.5 mm/s–4.5 mm/s and is approximately −1 mm/s–2 mm/s with the algorithm during the movement of the lower module. The result of the displacement error is shown (see Figure 13). The error without the algorithm is approximately −2.5 mm–1 mm and is approximately −1 mm–0.5 mm with the algorithm during the movement of the upper module. The error without the algorithm is approximately −1.5 mm–1 mm and is approximately −1 mm–0.5 mm with the algorithm during the movement of the lower module. In summary, the synchronous control algorithm significantly reduces errors and improves the stability of the device.

## 5. Conclusions and Future Work

This paper proposed a novel patient transfer assist system named E-pat-plus, which can be used for contactless transfer of patients in emergency medical situations such as COVID-19, thereby reducing the risk of infection and physical burden on caregivers. E-pat-plus transfers patients through the cooperative movement of a two-layer module structure. Regarding the mechanical design, a five-gear assembly module with limit blocks and a synchronous belt pulley set are presented; among them, the five-gear assembly module can drive the belt on both sides by only one motor, reducing the cost and complexity of the electronic control system. The flat synchronous belt pulley set has significant engineering implications; it effectively reduces the accumulation of thickness during belt winding on the rollers and prevents slippage and runout problems. For the control strategy, a cross-coupling control strategy based on fuzzy PID control suitable to the operating conditions was selected by comparison with the possible methods. Furthermore, the motion process of E-pat-plus was elaborated, and some preliminary experiments related to system performance, including load-bearing experiments and error experiments, were carried out, which verified the rationality and effectiveness of the device. It is worth mentioning that there are some shortcomings in the prototype for the current version. For example, to ensure the stability of the mechanical structure, all materials are made of aluminum alloy or stainless steel, which leads to a heavy weight of the device. In an emergency, it may be difficult for caregivers, especially females, to move the equipment. As another example, the synchronization control algorithm is separately applied to the upper and lower modules, and the control method between the upper and lower modules has not yet been completed, which may be one of the reasons for the discomfort of the patient.

In future work, further optimization work will be carried out, including mechanical structure and control algorithms. First, for noncritical load-bearing components, lightweight 3D printing materials (such as nylon, resin, etc.) can be used to reduce the total weight of the device. Second, some advanced synchronous control strategies, such as adaptive control and sliding mode control, need to be explored, and they may have better application effects on this device. Third, some sensors such as distance sensors and pressure sensors can be added to the system. The preliminary idea is that a distance sensor on the side of the equipment can detect whether the equipment is interfering with the stretcher/bed, and a pressure sensor on the surface of the equipment can be used as a switch to start the equipment to ensure the safety of movement. Finally, in order to apply E-pat-plus to real clinical scenes, the stability of the device under extreme conditions needs to be further tested, such as the ultimate load-carrying capacity, electromagnetic compatibility under severe electromagnetic field interference, etc. Generally, a prototype is provided and tested in this paper, and there is still much work to be done before commercialization.

## Figures and Tables

**Figure 1:** The prototype of E-pat-plus.

**Figure 2:** Working principle of E-pat-plus.

**Figure 3:** Configuration of the E-pat-plus.

**Figure 4:** Upper module of E-pat-plus. (a) Overview of the upper module and (b) five-gear assembly module.

**Figure 5:** Lower module of E-pat-plus.

**Figure 6:** Dynamic model of the upper module.

**Figure 7:** Comparison of the response value and errors of fuzzy PID and classic PID under a unit step signal.

**Figure 8:** Comparison of the simulation models of the three synchronization strategies.

**Figure 9:** Comparison of synchronization speed/displacement errors of three synchronization control strategies.

**Figure 10:** Transfer process of E-pat-plus. (a) Approaching the patient, (b) raising the patient, (c) human-machine integrated movement, and (d) completing the transit process.

**Figure 11:** Motor current of the (a) upper and (b) lower modules at the rated load.

**Figure 12:** Comparison of the speed error for conditions with/without the synchronous control strategy.

**Figure 13:** Comparison of the displacement error for conditions with/without the synchronous control strategy.

**Table 1:** Parameters in equation (4).

Number	Symbols	Implication	Unit
1	*T*_*m*_	Motor driving torque	N·m
2	*J*_*s*_	Rotational inertia of the motor and reducer	kg·m^2^
3	*B*_*s*_	Motor damping coefficient	—
4	*T*_*i*_	Output torque of driving gear *i*	N·m
5	*T*_*xi*_	Driving torque of the universal joint *i*	N·m
6	*J*_*xi*_	Rotational inertia of universal joint *i*	kg·m^2^
7	*J*_*pi*_	Rotational inertia of the roller *i*	kg·m^2^
8	*θ*_*mi*_	Rotation angle of driving gear *i*	rad/s
9	*θ*_*pi*_	Rotation angle of roller *i*	rad/s
10	*r*_*pi*_	Diameter of roller *i*	m
11	*μ*	Friction coefficient of flat belt	—
12	*m*_*i*_	Mass of human torso, head and feet	kg
13	*z*_*i*_	Number of teeth of gear *i*	—

## Data Availability

The data used to support the findings of this study are available from the corresponding author upon request.
